The article "A Narrative Review of Different Hemostatic Materials in Emergency Treatment of Trauma" was published in 2022. Journal: Emerg Med Int.

# A Narrative Review of Different Hemostatic Materials in Emergency Treatment of Trauma

**DOI:** 10.1155/2022/6023261

**Published:** 2022-10-21

**Authors:** Xiaoxiao Xiao, Zhoupeng Wu

**Affiliations:** ^1^West China Hospital Operation Room West China School of Nursing, Ichuan University, 37 GuoXue Alley, Chengdu 610041, Sichuan, China; ^2^Department of Vascular Surgery, West China Hospital, Sichuan University, 37 GuoXue Alley, Chengdu 610041, Sichuan, China

## Abstract

Hemostatic materials are very important for the treatment of a large number of bleeding trauma patients in battlefield and disaster environments. Different types of hemostatic materials need to be used for emergency hemostasis according to different injury parts and severity. At present, the first-aid hemostatic materials have been well applied to the bleeding of body surface wounds, limbs, and junctions, but there are still no ideal hemostatic materials in the early treatment of first aid for the deep and incompressible bleeding of thoracoabdominal cavity and visceral organs. This paper reviews the classification and mechanism of hemostatic materials, as well as the application and research progress in trauma emergency, so as to provide reference for the application of hemostatic materials in early first-aid emergency.

## 1. Introduction

Massive blood loss is one of the main causes of death caused by war and disaster accidents. 80% of the deaths of patients occur within 1 hour after trauma. If the bleeding can be stopped immediately or early, the mortality can be reduced to 20%∼30% [1]. For emergency trauma bleeding, the early hemostatic methods are usually to use hemostatic instruments, such as tourniquets and hemostatic forceps. [2, 3], to achieve hemostatic effect by compressing and closing the wound, but these methods may lead to secondary damage to the body, local tissue necrosis, and secondary infection [4–6]. In recent years, hemostatic materials reported at home and abroad include fibrin glue, polysaccharide, oxidized cellulose, and other new medical materials in addition to commonly used gauze, bandage, gelatin sponge, and zeolite. However, there is still a relative lack of hemostatic materials that can be applied to early trauma first aid in the world, and the mechanism of action of various hemostatic materials has not been fully clarified. There is a lack of relevant guidance materials on early trauma first aid [7]. In addition, the proportion of bleeding in various parts of trauma patients is 67% in the trunk, 19% in the junction parts such as the groin, armpit, and neck, and 14% in the limbs [8]. For trauma bleeding, it occurs in the trunk, and the bleeding in this part, such as internal bleeding involving important organs such as the heart, liver, and spleen, will cause a large amount of blood loss in a short time, causing hemorrhagic shock [9]. However, there is still no ideal first-aid hemostatic material for these incompressible bleeding.

## 2. Methods

In order to understand the application and research progress of different types of hemostatic materials in trauma first aid, we searched MEDLINE, CINAHL, EMBASE, AMED, ProQuest Hospital Collection, NHS Healthcare Databases Advanced Search to search AMED, British Nursing Index, CINAHL, EMBASE.HMIC, PsycINFO, Health Business Elite with “hemostatic material,” “hemostatic hydrogel,” “hemostatic dressing,” and “hemostatic powder” as keywords. The search period is from January 2005 to August 2022. The literature inclusion criteria are as follows: (1) the research object is hemostatic materials for first aid; (2) the research objects are hemostatic materials for clinical use and newly developed hemostatic materials of various types, with emphasis on hemostatic materials suitable for noncompressible blood loss; (3) the literature types are articles and reviews. The literature exclusion criteria are as follows: (1) literature with duplicate or obsolete content; (2) lectures and comments. Finally, 40 papers were included. We reviewed the classification and mechanism of existing hemostatic materials, as well as the application and research progress in trauma first aid, so as to provide reference for the application of hemostatic materials in early trauma first aid.

## 3. Result

There are many kinds of hemostatic materials [10–17], which can be divided into patch type (including gauze, nonwoven fabric, filaments, sponges, and membranes), particle powder type (including mineral hemostatic particles and hemostatic powders), fluid sealing type (including biological glue, chemical glue, wax, and liquid foam), and tactile expansion type (including compressed cotton and solid glue). The hemostatic materials shall have the characteristics of rapid hemostasis, no allergen, nontoxic degradation products, and can be absorbed by human body. Absorbable materials include gelatin, collagen, and chitosan from animals; oxidized cellulose, regenerated oxidized cellulose, and starch polysaccharide polymer from plants, and synthetic chemical colloids. In order to cope with the complex and diverse clinical bleeding situations, absorbable hemostatic materials have evolved into various forms to meet the hemostatic needs of different surgical wounds. For example, absorbable hemostatic materials mainly made of regenerated oxidized cellulose have developed many forms such as fibril, nonwoven cloth, and powder from the earliest form of gauze. Absorbable hemostatic materials with gelatin as the main material have developed from sponge to gelatin powder, and then to flowing gelatin matrix mixture. Absorbable hemostatic materials mainly made of collagen have developed from powder, sponge, and nonwoven cloth. The morphological characteristics of hemostatic materials determine their applicable wound types, functions, and effects. For example, sponges are soft and porous, absorbing liquid to expand, and suitable for tamping and pressing wounds to stop bleeding. Filaments are easy to be layered and shaped, suitable for large and irregular wound bleeding. Nonwoven fabrics have morphological memory and strong toughness, which are suitable for minimally invasive surgery wound bleeding. The powder is fine and granular, which can adhere to and disperse the wound surface. Fluids have fluidity and plasticity, which can penetrate into the cavity and stick to the wound surface and are suitable for hemostasis in complex cavities that are difficult to reach. Waxes are mainly used for bone wound bleeding. Hemostatic materials with the same material but different shapes have significant differences in hemostatic effects. For example, compared with ordinary gauze, nonwoven fabrics made of regenerated oxidized cellulose can shorten the hemostatic time by about 40%. The contact area of bleeding wound of fluid hemostatic materials made of gelatin is 98.1%, which is much higher than that of sponge (23.9%) [15–18]. The high contact rate of wound brings about the improvement of the hemostatic effect. Some studies have shown that fluid hemostatic materials have less bleeding than sponge hemostatic materials in spinal surgery. All of these hemostatic materials feature in Table 1.

### 3.1. Patch Type

Patch hemostatic materials are a kind of sheet-like materials that cover wounds, adhere to bleeding sites, and prevent further damage. The main hemostatic mechanism of patch hemostatic materials is to close the wound by fitting and covering with the damaged tissue, exert certain pressure on the wound, and form an effective physical barrier, and then use its internal pore structure to quickly absorb blood and water, activate the rapid aggregation of platelets, so as to achieve the hemostatic effect [11, 12] (Figure 1). The patch type hemostatic material is easy to use, can cover the wound quickly, and is well used in the body surface pressing wound. Currently, hemostatic patches in clinical use include hemostatic gauze, chitosan dressing (hemcon), and collagen sponge (gelfix). Hemcon is a hemostatic sheet made by freeze-drying chitosan acetic acid solution. It has good hemostatic effect and has been used in military medical treatment in the United States. However, its disadvantage is that its freeze-drying molding process makes the product hard, and the effect of the material fitting the wound is poor. It needs external force to achieve better hemostatic effect [17]. Gelfix has good fitting performance. Its main component is collagen extracted from bovine Achilles tendon. Collagen is mixed with other materials as matrix material and prepared through defoaming, curing, freeze-drying, and sterilization [6]. Collagen can stimulate platelet aggregation and adhesion at the injured site, generate fibrin, form thrombus, and stop bleeding, but it has been reported that its toughness is poor and is not conducive to wound healing [18, 19]. In recent years, the research on patch hemostatic materials mainly focuses on enhancing their adhesion to improve the hemostatic effect in emergency environments. Li et al. [20] developed an elastic adhesive hemostatic material (TA) with strong adhesion on various wet surfaces. TA is composed of a positively charged adhesive layer and an alginate polyacrylamide matrix layer. The adhesive layer adheres to the tissue through electrostatic action. The matrix layer dissipates energy to ensure the stability of the material. At the same time, alginate endows it with hemostatic ability. Therefore, Ta has been proven to be used for immediate hemostasis and efficient sealing of wounds on wet surfaces of organs. Gao et al. [21] developed a hydrogel composite patch (HMC). They redeveloped the medical patch that has been used at present, and recrosslinked it with the hydrogel with good adhesion, forming a topological interpenetrating network structure with strong adhesion, which effectively overcomes the shortcomings of poor adhesion of medical patches. Experiments have shown that under the impact of large pressure blood flow, HMC in the sheep common carotid artery blood loss model and liver blood loss model can achieve no deformation and no shedding, fit well on the wound surface, and close the wound to achieve a good hemostatic effect [21]. In recent years, the adhesive properties of patch hemostatic materials have been continuously enhanced, and they have gradually got rid of the assistance of external pressure. However, further research and development of materials that can be rapidly degraded or noninvasive peeled are needed.

### 3.2. Granular Powder Type

Granular powder hemostatic materials are also a kind of materials that have been studied earlier, usually small particle size materials obtained by grinding and freeze-drying after raw materials are synthesized. The granular powder hemostatic material can better cover wounds of different shapes and depths. Its mechanism of action mainly relies on the small particle structure of hemostatic powder to absorb water in blood, effectively concentrate blood, closely adhere to damaged tissues under the action of external forces, and electrostatically interact with negatively charged red blood cells with the help of some self-positively charged components such as chitosan, so as to promote the formation of local blood clots and accelerate hemostasis [13] (Figure 2).

Because of its convenient use and strong shape plasticity, granular powder hemostatic materials are suitable for large and deep body surface wounds or on-site emergency hemostasis with limited treatment conditions. At present, granular powder materials in use include zeolite, microfibril collagen powder (MFC), and chitosan hemostatic powder (celox). Zeolite has excellent adsorption capacity due to its high specific surface area. It can quickly adsorb blood after contacting with wounds and promote blood coagulation through exothermic action. It is well used in emergency hemostasis of battlefield body surface injury, but high temperature may cause damage to damaged tissues [22]. The main component of MFC is bovine collagen, which is easy to adhere to bleeding wounds and can promote platelet aggregation on the surface of materials, so as to quickly stop bleeding [23]. This material has certain biodegradability, but because it contains foreign proteins, the residual foreign proteins after degradation may cause granulation swelling and infection in the wound, which usually requires later surgical removal [24, 25]. Celox is the third-generation hemostatic product of the U.S. military. The main component is chitosan [8], which can quickly control the bleeding of the large artery caused by trauma and will not produce heat and burn [26]. The existing granular powder hemostatic materials are mainly used for first-aid hemostasis with limited conditions and are suitable for wounds with small blood loss but irregular shape. The characteristics of powder particle materials that can quickly fill wounds can be used for emergency hemostasis, but it is often difficult to achieve ideal results for large wounds with large blood loss. In recent years, some biodegradable granular powder hemostatic materials have been developed one after another. Huang et al. [27] prepared a biodegradable granular hemostatic composite (SACC) composed of sodium alginate, carboxymethyl chitosan, and collagen through emulsification and cross linking. SACC has uniform spherical structure, rough surface, and good water absorption, which enhance its hemostatic ability. The results of coagulation experiments in vitro and hemostasis experiments in vivo in rats show that SACC has better hemostatic effect than chitosan and sodium alginate alone. At the same time, the fluorescence labeling experiment confirmed that SACC has good biodegradability [27]. At present, more attention has been paid to controlling the dosage of granular powder materials and increasing their rapid degradation ability. The latest granular powder type hemostatic products and methods include Combat Gauze (ZMedica Corporation, Wallingford, CT, USA; http://www. z-medica.com/), Celox gauze (Medtrade Products Ltd., Crewe, UK; http://www.celoxmedical.com/usa/products/celox-gauze/), and ChitoGauze (HemCon Medical Technologies, Portland, OR, USA; http://www.hemcon.com/). These hemostatic dressings have been recommended in the US military Tactical Combat Casualty Care guidelines and have been covered in a recent systematic review.

### 3.3. Fluid Seal Type

Fluid sealing hemostatic materials are new materials that have emerged in recent years. These materials are usually stored in the form of liquid. After contacting the wound by local injection/spraying, they form glue or film to close the wound. Its mechanism of action mainly relies on the high adhesion of the material to closely combine with the damaged tissue and close the wound. While forming a physical barrier, it uses some components that can promote the aggregation of red blood cells and platelets to accelerate hemostasis [14–16] (Figure 3).

Fluid sealing hemostatic materials are suitable for deep and irregular wound bleeding in the body due to their high fluidity and adhesion, especially for uncontrollable wound bleeding such as internal defect bleeding of the organs and bones. Clinically used fluid sealing hemostatic materials such as cyanoacrylate tissue adhesive are often used for puncture wound bleeding in the cavity. It can react anionically with the water in the tissue or blood and solidify into glue to seal the wound, so as to achieve the rapid hemostatic effect, but it will lead to a certain degree of inflammation and tissue necrosis [28, 29]. Hemostatic materials prepared based on chemical synthetic substances often have poor biocompatibility. Therefore, hemostatic materials prepared from natural substances have been developed one after another, such as fibrin glue (FS). FS is a kind of biological hemostatic material extracted from human plasma, mainly composed of thrombin, fibrinogen, and other preparations. It can imitate the process of fibrinogen forming fibrin monomer under the action of thrombin and calcium ion in the coagulation process, and finally form stable blood clot to achieve the hemostatic effect [30]. It is often used for hemostasis of the organs in abdominal surgery, but this material leads to serious postoperative adhesion [31, 32]. Hong et al. [33] prepared a matrix gel that mimics the extracellular matrix. The material is mainly composed of gelatin modified by methyl methacrylate and hyaluronic acid modified by o-nitrobenzyl light trigger molecules. They injected matrix gel's gel solution into the bleeding hole in the pig's heart through a syringe. After irradiating the wound with ultraviolet rays, the gel solution quickly gelled and fixed, and the bleeding stopped within 10 s. Continuous observation after operation found that the material had good adhesion on the wet dynamic surface [33]. At the same time, the material has good biocompatibility, so the wound healing effect is better after operation. There are also some hemostatic materials that can be quickly degraded after surgery on the basis of immediate hemostasis, which is conducive to later healing. For example, Huang et al. [34] developed an absorbable hemostatic hydrogel (chi-c/dacnc) suitable for noncompressible bleeding, which can be injected into deep and irregular bleeding parts and bone defect areas, quickly self-healing synthetic glue and completely filling the defect parts to achieve the hemostatic effect. At the same time, it has the ability of rapid biodegradation and is conducive to wound healing. Due to its high adhesiveness, this kind of material is easy to cause adhesion of surrounding tissues after local use,and may cause intestinal obstruction in severe cases, requiring secondary surgery. Therefore, in the process of research and development, this kind of material should be considered to both seal the wound and prevent adhesion. The representation of flowable hemostatic agents is the dry fibrin sealant powder called Fibrocaps (Raplixa; ProFibrix BV, Leiden, Netherlands) [35, 36]. The product is provided in 1 g in a vial and is easy to use and store. It consists of 79 mg of human plasma-derived fibrinogen and 726 U of human plasma-derived thrombin that has been separately spray-dried with trehalose to produce soluble, free-flowing microparticles. Intracavitary foam is based on a fibrin sealant embedded in a biomimetic complex polymer [37]. The so-called ClotFoam is a gelatin-based hydrogel carrying a fibrin monomer and produced from a mixture of four liquid components (e.g., gelatin, transglutaminase enzyme, fibrin monomer, and factor XIII) [38–42]. It is currently an investigational product under phase 1 clinical trial for hemostasis in liver bleeding [43].

### 3.4. Trigger Expansion Type

Trigger inflation hemostatic materials are also a research hotspot in recent years. These materials usually have macroporous structure and shape memory function. Its mechanism of action is mainly through the unique shape memory macroporous structure of the material to highly fit the size of the wound and quickly absorb blood and water, effectively seal the bleeding position and promote coagulation(Figure 4).

Trigger inflation hemostatic material has the characteristics of rapid expansion and strong water absorption, which is very suitable for hemostasis of large noncompressible wounds. It has great application potential in the hemostatic direction of penetrating wound bleeding at the junction of the trunk [35, 36, 44]. This kind of representative hemostatic material used clinically, such as the cellulose hemostatic sponge (xstat) used by the US military, is compressed to a small volume through extrusion after synthesis, and can expand to its original size after being triggered by water or blood, quickly absorb blood and close wounds, so as to achieve hemostatic effect. The latest XStat (Revmedx, Wilsonville, OR, USA) is composed of a multitude of rapidly expanding minisponges loaded in a syringe. It can be injected into deep wounds, then quickly expands and creates an internal compression to achieve hemostasis. The sponges are not biodegradable and need to be removed, and each has a tiny radiopaque marker so that any remaining in the body can be spotted on *X*-ray [45]. This material is mainly used in the battlefield for bleeding at the junction of the trunk and limbs where hemostasis cannot be pressed [37, 38]. This kind of hemostatic material is relatively novel, which can effectively stop bleeding and protect wounds for ballistic penetrating wounds at the junction. However, at present, this kind of material has a single function, which is not suitable for hemostasis in thoracoabdominal, sacrum, clavicle, and other parts, and needs to be removed during definitive surgery. Wang et al. [39] synthesized a self-expandable porous composite (Cmcp) that can be adaptively adjusted according to the shape of the wound by using carboxymethyl cellulose fiber and acetaldehyded polyvinyl alcohol. The fiber porous network structure and strong water absorption endow the material with liquid triggered self-expansion ability, and at the same time, it can achieve shape adjustment in wounds of different depths and shapes, so as to fill the wounds quickly and fully, which is suitable for fatal bleeding in larger wounds. In the pig model of femoral artery massive hemorrhage, Cmcp expands rapidly after contacting with the wound, rapidly absorbs blood through its fibrous porous network structure, activates platelets and coagulation factors to quickly form thrombus, and achieves hemostatic effect [39]. At the same time, the results of CT scanning and three-dimensional reconstruction show that Cmcp can completely fit the wound site through its shape adaptability, playing a role of sealing and protection, which is conducive to wound repair. In the later research, it can be considered to endow the material with antibacterial, anti-inflammatory, and wound healing functions on the basis of rapid hemostasis.

## 4. Conclusion and Prospect

Rapid hemostasis in trauma first aid has always been the focus of medical attention at home and abroad, and the related research of various hemostatic materials has also increased year-by-year. Based on the difference of the external morphology of the existing hemostatic materials, the author divides them into patch type, particle powder type, fluid sealing type, and trigger expansion type, and analyzes and summarizes the hemostatic mechanism, application scenarios, and research status of each type of hemostatic materials. Based on the above analysis, the hemostatic mechanism of these hemostatic materials includes forming a physical barrier with the wound to close the wound, absorbing the blood and water of the wound, promoting the aggregation of red blood cells and platelets, and accelerating the coagulation process. Different types of hemostatic materials have their own characteristics in hemostatic mechanism, such as high-strength wound coverage of patch type, small particle size structure of particle powder type fitting blood loss point, gel forming and film forming characteristics of fluid seal type, and shape memory function of trigger expansion type. Different types of hemostatic materials are suitable for different trauma situations in trauma emergency treatment because of their respective characteristics and advantages and disadvantages. Patch hemostatic materials are suitable for bleeding from wounds on the surface of the body and organs due to their strong adhesion and high coverage. The granular powder hemostatic material is suitable for emergency hemostasis of small blood loss and irregular shape because of its small particle size and easy to fill wounds. Because of its high fluidity and strong adhesion, the fluid sealed hemostatic material can highly fit the wound and play an effective sealing role, which is suitable for blood loss in noncompressible wounds such as deep wound and organ and bone damage. The rapid shape adaptation of trigger inflation hemostatic materials endows them with the ability to cope with uncompressed bleeding, which is especially suitable for penetrating injuries and massive blood loss at the junction of the limbs and trunk. Therefore, in trauma first aid, suitable hemostatic materials and methods should be selected according to the injured site and bleeding characteristics.

In addition, wound infection and secondary multiple organ dysfunction are the causes of the third wave of death peak after trauma. The repair of the wound tissue is a dynamic and multistage process. The author believes that ideal first-aid hemostatic materials should have antibacterial, repair promoting, degradable, and other characteristics, and can respond intelligently according to the physiological microenvironment of the wound (such as temperature and pH changes). For noncompressible bleeding such as abdominal bleeding, in addition to developing targeted hemostatic materials, we should also study intelligent, portable, and miniaturized diagnosis and treatment equipment that can be used on-site. For example, intelligent blood transfusion equipment, intelligent hemostasis equipment integrating accurate diagnosis and laparoscopy, intelligent life monitoring and support system, etc. will significantly improve the efficiency and level of on-site treatment of trauma patients.

None of the current hemostatic products meet all the criteria for an ideal hemostatic agent. There is still a tremendous impetus for the development of diverse and more efficacious hemostatic technologies and biomaterials for emergency scenarios, not only in both civilian and military traumatic settings but also during variable therapeutic interventions. Alternatively, large randomized trials, particularly direct head-to-head clinical trials comparing the current hemostatic agents, are needed to show which is more effective in prehospital hemorrhage control. There is also a need for studies that would enable the selection of appropriate hemostatic agents based on the mechanism and location of injuries. Finally, nanotechnology has been applied for hemostasis [46]. Some novel hemostatic agents based on nanomaterials are intriguing [47]; however, it may be some time before they are brought to clinical trials. For example, nano- and micromaterials have been developed for the treatment of internal bleeding and uncontrolled hemorrhage [48]; however, these novel hemostatic agents again may prove to be efficacious (or not) with further studies. There are also new delivery systems (e.g., self-driven and trauma-targeted delivery) that would make current hemostatic agents more effective [43, 45–49].

## Figures and Tables

**Figure 1:** By attaching and covering the damaged tissue to close the wound, there is a certain pressure effect on the wound and form an effective physical barrier, and then use its internal pore structure to quickly absorb blood and water, activate platelets to accumulate quickly, and achieve the effect of hemostasis.

**Figure 2:** The small particle structure of hemostatic powder absorbs the water in the blood, effectively concentrates the blood, and closely fits with the damaged tissue under the action of external forces, while with the help of some positively charged components such as chitosan, electrostatic effect occurs with negatively charged red blood cells, prompting the local formation of blood clots to accelerate hemostasis.

**Figure 3:** Relying on the high adhesion of the material to closely bind to the damaged tissue and close the wound, while forming a physical barrier, using some components that can promote the aggregation of red blood cells and platelets to accelerate hemostasis.

**Figure 4:** Through the material's unique shape-memory large pore structure, it highly fits the size of the wound and quickly absorbs blood and water, effectively blocking the bleeding location and promoting coagulation.

**Table 1:** Features of various hemostatic materials.

Types	Mechanisms	Indications	Products
Patch	By attaching and covering the damaged tissue to close the wound, there is a certain pressure effect on the wound and form an effective physical barrier, and then use its internal pore structure to quickly absorb blood and water, activate platelets to accumulate quickly, and achieve the effect of hemostasis	Suitable for bleeding from wounds on the surface of the body and organs and used in battlefield and prehospital environments	Battle gauze (NATO use), chitosan dressings (Chito Gauze, Celox gauze), and collagen sponges (Gelfix)

Granular powder	The small particle structure of hemostatic powder absorbs the water in the blood, effectively concentrates the blood, and closely fits with the damaged tissue under the action of external forces, while with the help of some positively charged components such as chitosan, electrostatic effect occurs with negatively charged red blood cells, prompting the local formation of blood clots to accelerate hemostasis	Suitable for large, deep surface wounds or on-site emergency hemostasis with limited treatment conditions	Kaolin, zeolite, microfiber collagen powder (MFC), chitosan hemostatic powder (Celox), and rhombus zeolite gel particles

Fluid seal	Relying on the high adhesion of the material to closely bind to the damaged tissue and close the wound, while forming a physical barrier, using some components that can promote the aggregation of red blood cells and platelets to accelerate hemostasis	It is suitable for deep and irregular wound bleeding in the body, especially noncompressible wound bleeding such as organ and bone internal lack of blood loss	Cyanoacrylate tissue adhesive, Fibrin gum (FS), Matrix Gel, absorbable hemostatic hydrogel (CHI–C/DACNC)

Trigger expansion	Through the material's unique shape-memory large pore structure, it highly fits the size of the wound and quickly absorbs blood and water, effectively blocking the bleeding location and promoting coagulation	Hemostasis of large noncompressible wounds as an adjunct to the treatment of junction bleeding (i.e., neck, armpit, and inguinal bleeding).	XStat, self-expanding porous composites (CMCP)
